# A Meta-Analysis of the Effect of Exercise Rehabilitation Care on Cardiac Function in Patients with Chronic Heart Failure

**DOI:** 10.1155/2022/2507680

**Published:** 2022-07-04

**Authors:** Dawei Lv

**Affiliations:** Outpatient Department, The Fourth Medical Center of Beijing People's Liberation Army General Hospital, Beijing 100048, China

## Abstract

**Aims:**

Effect of systematic exercise rehabilitation nursing on patients with chronic heart failure.

**Materials and Methods:**

From January 1, 2021, to March 22, 2006, a comprehensive search was conducted on China Knowledge Network (CNKI), Wanfang, VIPERS (VIP), China Biomedical Literature Database (CBM), PubMed, Cochrane Library, EMBASE library database, and clinical registry to obtain the literature on the impact of exercise rehabilitation nursing on cardiac function of patients with chronic heart failure. From January 1, 2006, to March 22, 2021, the literature of randomized controlled trials (RCTs) on the effect of exercise rehabilitation nursing on cardiac function in patients with chronic heart failure was collected. According to the inclusion and exclusion criteria, literature screening, data extraction, and quality evaluation were carried out. Cochrane system assessor manual version 5.0 was used for quality assessment, and Review Manager Version 5.3 was used for meta-analysis.

**Results:**

A total of 9 articles were included, including 752 patients. Meta-analysis showed that exercise rehabilitation nursing had a significant effect on cardiac function indexes (LVESV, LVEF, CRP, BNP, and LVEDV) in patients with chronic heart failure (*P* < 0.05).

**Conclusion:**

Exercise rehabilitation nursing has a good effect on improving cardiac function in patients with chronic heart failure. It can improve cardiac function indexes such as left ventricular end-systolic volume, right ventricular ejection fraction, brain natriuretic peptide, and left ventricular end-diastolic volume in patients with chronic heart failure.

## 1. Introduction

Chronic heart failure refers to myocardial injury caused by hemodynamic overload, myocardial infarction, and cardiomyopathy, which leads to changes in myocardial structure and function and finally to poor cardiac pumping or filling function, accounting for about 20% of heart diseases in the same period, while mortality accounts for 40% of heart diseases in the same period [1, 2]. With the change in health concept, the goal of chronic heart failure is not only to save lives and improve organ function but also to improve patients' cardiac function and return to family and society as soon as possible [3]. Exercise rehabilitation nursing is very beneficial to the rehabilitation of chronic heart failure patients. It has obvious advantages such as shortening hospitalization time, reducing hospitalization rate, and increasing walking distance and can improve the psychological state and quality of life of patients [4]. Traditional nursing care for patients with heart failure involves absolute bed rest when treating and nursing heart failure. Exercise rehabilitation has changed the limitation that patients with heart failure can only be treated with drugs alone [5]. While achieving good treatment and nursing effects, it also puts forward a new research direction for the nursing of chronic heart failure [6]. Exercise rehabilitation nursing can promote the early rehabilitation of patients with chronic heart failure and improve their postoperative cardiac function, but there are still potential safety hazards in practice [7]. Therefore, this study conducted a meta-analysis of the published randomized controlled trial (RCT) literature on the effect of exercise rehabilitation nursing on cardiac function in patients with chronic heart failure in order to provide evidence-based medical evidence for clinical nursing care of the disease.

## 2. Materials and Methods

### 2.1. Inclusion and Exclusion Criteria

#### 2.1.1. Inclusion Criteria

The inclusion criteria were as follows: ① research type: the type of published literature must be collected based on RCTs regardless of whether the method is blinded or not, and the language is limited to Chinese and English; ② in line with the relevant judgments of chronic heart failure, their gender, race, body mass index, and disease course are not limited; ③ intervention measures: the intervention measures in the observation group are exercise rehabilitation nursing or rehabilitation exercise training, and the control group adopts routine nursing and other measures; the number of cases was more than 20; ④ outcome indicators: the selected outcome indicators included the literature with cardiac function as the main evaluation and research indicator.

#### 2.1.2. Exclusion Criteria

The exclusion criteria were as follows: ① the type of study did not clearly describe the randomized controlled trial; ② the effective outcome data could not be extracted from the literature; ③ the paper was published repeatedly; ④ the full text could not be obtained; F06E patients had other cardiac diseases such as conduction block and hematopoietic system diseases; ⑥ the sample size is too small.

### 2.2. Retrieval Strategy

The documents retrieved this time are published randomized controlled trials of the application of exercise rehabilitation nursing on cardiac function in patients with chronic heart failure. Through computer retrieval, China National Knowledge Infrastructure (CNKI), Wanfang, VIP (VIP), China Biomedical Literature Database (CBM), PubMed, Cochrane Library, Embase Library database, and clinical registries were searched to obtain the literature. The search period was from January 1, 2006, to March 22, 2021, and references in the included literature were tracked and included in relevant studies where possible. The Chinese search terms are as follows: ① disease type: “chronic heart failure” or “chronic heart failure” or “chronic heart failure” or “chronic heart failure” or “chronic heart failure” or “chronic congestive heart failure”; ② intervention measures: “exercise rehabilitation nursing” or “rehabilitation nursing”; ③ research method: “randomized control” or “randomized” or “ROT.” The English search terms are based on the characteristics of each database by combining the corresponding subject headings and keywords for retrieval, and duplicate documents are eliminated. The English search terms are as follows: ① disease type: “chronic heart failure” OR “chronic heart failure” OR “chronic heart failure” OR “chronic heart failure” OR “chronic heart failure” OR “chronic congestive heart failure”; ② intervention measures: “sports rehabilitation care” OR “Rehabilitation Care”; ③ Research method: “ROT” OR “Randomized control.”

### 2.3. Literature Screening and Quality Evaluation

After the literature search was completed, two reviewers independently screened the literature, first read the literature titles, abstracts, and other information, and excluded obviously unqualified literature (such as reviews and animal experiments). Then, according to the inclusion and exclusion criteria, the unqualified literature (such as self-controlled trials) was further excluded. Three screenings included the following: reading the full text carefully and excluding the literature with unclear outcomes and diagnoses. If the valid information provided in the article is unclear or missing, it is necessary to contact the author by phone, e-mail, etc. to obtain relevant information. When two reviewers disagree on whether to include the article, they should consult an expert to resolve it. All included studies were evaluated according to the Cochrane Manual of Systematic Review, and publication bias was represented by a funnel plot.

### 2.4. Statistical Methods

Meta-analysis was performed using RevMan5.2 software provided by Cochrane Collaboration. The *χ*2 test was used for the statistical heterogeneity test. If the result was *P* ≥ 0.10 and I^2^ ≤ 50%, it indicated that there was no significant heterogeneity between the observation groups, and the fixed-effect model was used to describe the data; if the heterogeneity test result was *P* < 0.10 and I^2^ > 50%, it indicated that there is heterogeneity between groups; the source of heterogeneity is investigated, and subgroup analysis or sensitivity analysis was performed on the results. The final homogeneity uses a fixed-effect model. For qualitative analysis, a random-effect model was used to combine effect values, and descriptive analysis was used for the literature that was not suitable for inclusion in meta-analysis. The measurement data of continuous variables were expressed by the weighted mean difference (WMD) and its 95% confidence interval, and *P* < 0.05 was considered to be statistically significant.

## 3. Results

### 3.1. Literature Search Results

After database retrieval, 479 articles were initially detected, including 65 articles from CNKI, 115 articles from Wanfang, 153 articles from VIP, 89 articles from PubMed, and 57 articles from other databases. After strict screening according to the inclusion and exclusion criteria, 9 studies were finally included, as shown in Figure 1.

### 3.2. Basic Information of Included Studies

A total of 9 articles were included, including a total of 752 patients, of which 385 patients in the observation group received exercise rehabilitation nursing and 367 patients in the control group received routine nursing, and the nursing time was 14 days to 6 months. Nine studies had clear diagnostic criteria; all nine studies had a balanced baseline (Table 1).

### 3.3. Methodology and Risk of Bias Assessment of Included Studies

The risk of bias assessment of the included studies was assessed and described according to the risk of bias assessment tool recommended by the Cochrane Handbook for methodological bias assessment of the included studies (Figures 2 and 3).

### 3.4. Inclusion of Literature-Related Indexes of Cardiac Function

The quality of the literature in this study was scored on the BSHS-A, including the left ventricular end-systolic volume (LVESV), right ventricular ejection fraction (LVEF), C-reactive protein (CRP), brain natriuretic peptide (BNP), and left ventricular end-diastolic volume (LVEDV) scores for each dimension (Table 2).

### 3.5. Meta-Subgroup Analysis Results

#### 3.5.1. Left Ventricular End-Systolic Volume Changes after Care in Both Groups

In the study, a total of 9 publications reported general health status. On the test of heterogeneity, Q-test with *P* > 0.05 and I^2^ = 37% < 50% indicated that the included studies were homogeneous. Sensitivity analysis was performed on the current nine studies, and none of them caused significant interference with the results of this meta-analysis, implying that this study has good stability. Therefore, a fixed-effects model was used for the analysis, and the results showed that *Z* = 7.90 and *P* < 0.0001, a statistically significant difference, indicating that exercise rehabilitation care was effective in improving left ventricular end-systolic volume in patients with chronic heart failure. The presence of publication bias in this study was examined by plotting a funnel plot, which was symmetrical, implying no publication bias (Figure 4).

#### 3.5.2. Changes in Right Ventricular Ejection Fraction after Care in Both Groups

Nine studies reported general health status in the literature. On the test of heterogeneity, Q-test with *P* > 0.05 and I^2^ = 12% < 50% indicated homogeneity of the included studies. Sensitivity analysis was performed on the current nine studies, and none of them caused significant interference with the results of this meta-analysis, implying that this study has good stability. Therefore, a fixed-effects model was used for the analysis, and the results showed that *Z* = 10.42 and *P* < 0.0001, a statistically significant difference, indicating that exercise rehabilitation care is effective in improving right ventricular ejection fraction in cardiac function in patients with chronic heart failure. The presence of publication bias in this study was examined by plotting a funnel plot, which was symmetrical, implying no publication bias (Figure 5).

#### 3.5.3. Changes in C-Reactive Protein after Care in Both Groups

General health status was reported in the 9 papers of the study. On the test of heterogeneity, Q-test with *P* > 0.05 and I^2^ = 0% < 50% indicated homogeneity of the included studies. Sensitivity analysis was performed on the current nine literature studies, and none of them caused significant interference with the results of this meta-analysis, implying that this study has good stability. Therefore, a fixed-effects model was used for the analysis, and the results showed that *Z* = 15.59 and *P* < 0.0001, a statistically significant difference, indicating that exercise rehabilitation care is effective in improving C-reactive protein on cardiac function in patients with chronic heart failure. The presence of publication bias in this study was examined by plotting a funnel plot, which was symmetrical, implying no publication bias (Figure 6).

#### 3.5.4. Changes in Brain Natriuretic Peptide after Care in Both Groups

A total of nine papers in the study documented somatic function. On the test of heterogeneity, I^2^ = 36% > 50% and Q-test with *P* > 0.05 indicated the homogeneity of the included studies. Sensitivity analysis was performed on the current nine studies, and none of them caused significant interference with the results of this meta-analysis, implying that this study has good stability. Therefore, a fixed-effects model was used for the analysis, and the results showed a statistically significant difference of *Z* = 1.04, indicating that exercise rehabilitation care was effective in improving brain natriuretic peptide in patients with chronic heart failure on cardiac function. The presence of publication bias in this study was examined by plotting a funnel plot, and the symmetry of the funnel plot implies that there is no publication bias (Figure 7).

#### 3.5.5. Left Ventricular End-Diastolic Volume Changes after Care in Both Groups

The nine papers of this study, after the heterogeneity test, with I^2^ = 37% < 50% and *P*=0.12 > 0.1 for *Q* test, suggest that there is no heterogeneity between the papers selected for this study and fixed effects can be selected for meta-analysis. To ensure the accuracy and stability of the study, sensitivity analysis was continued. Sensitivity analysis was performed on the nine papers of this study, and none of them caused much interference with the results of this meta-analysis, implying that this study has good stability. The MD value of the nine studies pooled was −8.16, with a 95% confidence interval of 6.07 to 10.25, and was statistically significant, with *z* = 7.66 and *p*=0.000001 < 0.05, suggesting that exercise rehabilitation care was effective in improving left ventricular end-diastolic volume in patients with chronic heart failure (Figure 8).

## 4. Discussion

In recent years, the incidence rate of chronic heart failure has gradually increased and patients are prone to producing many negative emotions, such as anxiety and depression, which have a poor prognosis for patients' rehabilitation [8]. In addition, patients with chronic heart failure with long-term symptoms often need hospitalization, which increases the economic burden, makes them bear greater psychological pressure, and leads to more serious anxiety and depression [9]. Exercise rehabilitation nursing intervention can effectively improve the negative emotions of patients with chronic heart failure and improve the indexes of cardiac function to a certain extent [10]. The main reason for this situation may be that when facing the corresponding stress events, sports rehabilitation nursing is more likely to affect the patient's real thoughts, activate the cognitive system, lead to extreme and absolute wrong judgment and fear of death, lead to depression, and make them unable to cooperate properly with scientific sports rehabilitation nursing [11]. The implementation of sports rehabilitation nursing is to correct the cognitive distortion of patients, release the adverse psychological problems in psychology, completely eliminate the inner concerns of patients, find key problems, actively provide scientific and correct solutions, and improve the confidence in treatment so as to maintain the best mental state against diseases [12]. In addition to targeted drug therapy, scientific and effective nursing is the key to the treatment of patients with chronic heart failure. Traditional nursing mainly focuses on bed rest and sedation and limits exercise as much as possible, which not only leads to the decline of exercise ability but also leads to the formation of complications such as venous thrombosis and constipation, which seriously hinders the recovery of patients' conditions. In addition, with the popularization of exercise therapy in clinical practice, more and more clinical practice shows that exercise rehabilitation therapy can effectively improve the blood flow of skeletal muscle in patients with chronic heart failure, promote muscle contraction, and promote the metabolism of patients, so as to significantly improve their cardiac function and improve their quality of life.

In this study, an objective and systematic evaluation of the index efficacy of exercise rehabilitation care on cardiac function in patients with chronic heart failure was conducted by meta-analysis. The results found that a total of 9 papers including 848 patients were included, and the meta-analysis showed that the differences between the groups of exercise rehabilitation care on the indexes of cardiac function in patients with chronic heart failure were statistically significant. There are three main aspects of exercise rehabilitation care for cardiac function that can draw consensus among researchers: it can enhance the contractility of patients with chronic heart failure, improve their self-efficacy, and improve their quality of life [13]. Exercise rehabilitation care is the development of a care plan adapted to the patient's physical condition according to the severity of his condition, and by urging the patient to exercise effectively, it improves the body's hemodynamic indexes and optimizes cardiac function [14]. Exercise rehabilitation care helps patients to relieve tension, anxiety, and other negative emotions and motivates them. In addition, when implementing exercise rehabilitation care, attention is paid to the actual physical condition of patients with different levels of cardiac function, and a suitable exercise rehabilitation program is developed so that each patient can transition from passive to active exercise and make the whole program complete, which can effectively improve the clinical effect of treatment and improve cardiac function [15]. Exercise rehabilitation therapy can improve the dysfunction of peripheral vasodilatation and constriction by improving blood flow to the skeletal muscles [16].

Although this study was evaluated objectively, it still has shortcomings. The literature included in the study was small and the quality of the articles was low. The sample was estimated for only nine articles, and some articles had irregular random assignment methods, lacking allocation concealment, blinding, and review, with a high risk of bias [17].

In conclusion, exercise rehabilitation nursing can effectively improve the cardiac function of patients with chronic heart failure and improve the cardiac function indexes of patients with chronic heart failure, such as left ventricular end-systolic volume, right ventricular ejection fraction, brain natriuretic peptide, and left ventricular end-diastolic volume. However, the literature included in the evaluation had small sample size, small quantity, and insufficient quality. It is necessary to further expand the sample and high-quality RCR for in-depth and comprehensive scientific evaluation.

## Figures and Tables

**Figure 1:** The flow chart of literature screening.

**Figure 2:** Percentage of methodological quality assessment of the literature.

**Figure 3:** Literature bias risk assessment.

**Figure 4:** Meta-analysis of left ventricular end-systolic volume.

**Figure 5:** The meta-analysis graph of right ventricular ejection fraction.

**Figure 6:** Meta-analysis graph of C-reactive protein.

**Figure 7:** Plot of meta-analysis of brain natriuretic peptide.

**Figure 8:** Meta-analysis of left ventricular end-diastolic volume.

**Table 1:** Basic characteristics of the included literature.

Author	Year of publication	Research site	Sample size (test group/comparison group)	Age (years)	Gender (male/female)	Follow-up time (months)
[8]	2016	Shanghai	30/30	56.78 ± 4.32	30/30	6
[9]	2018	Henan province	57/57	63.43 ± 7.92	63/51	1
[10]	2016	Guangzhou city	40/40	56.30 ± 1.40	43/37	12
[11]	2017	Shenzhen	41/41	59.14 ± 10.88	45/37	6
[12]	2020	Shenzhen	49/49	64.60 ± 2.70	69/29	3
[2]	2017	Shaanxi province	40/40	71.3 ± 10.4	49/33	6
Bunny Pozehl	2015	United Kingdom	30/30	68.60 ± 8.50	35/25	3
[5]	2017	United States	61/60	64.3 ± 11.7	63/58	6
[1]	2019	Shandong	37/20	68.10 ± 1.14	41/16	3

**Table 2:** Relevant indexes of cardiac function in the included literature.

Author	Group	LVESV (mL)	LVEF (%)	CRP (/mmol/L)	BNP (pg/mL)	LVEDV (mL)
[8]	Comparison group	76.31 ± 13.51	43.23 ± 12.26	1.61 ± 0.41	375.74 ± 31.23	122.75 ± 21.26
	Observation group	67.30 ± 13.52	53.76 ± 11.15	1.30 ± 0.32	326.75 ± 31.22	111.34 ± 13.25

[9]	Comparison group	72.63 ± 12.32	42.75 ± 11.26	1.63 ± 0.32	372.97 ± 31.14	127.33 ± 12.24
	Observation group	69.62 ± 12.31	51.34 ± 13.25	1.22 ± 0.31	310.83 ± 32.10	116.30 ± 11.23

[10]	Comparison group	73.31 ± 12.81	47.33 ± 12.24	1.61 ± 0.81	371.34 ± 32.25	124.31 ± 22.81
	Observation group	61.30 ± 12.19	56.30 ± 11.23	1.30 ± 0.19	327.33 ± 31.24	114.30 ± 22.19

[11]	Comparison group	76.67 ± 13.24	46.30 ± 11.22	1.67 ± 0.24	367.23 ± 30.57	126.67 ± 23.24
	Observation group	63.23 ± 12.26	53.77 ± 11.14	1.23 ± 0.26	303.24 ± 31.25	113.23 ± 22.26

[12]	Comparison group	73.76 ± 21.15	47.37 ± 11.20	1.66 ± 0.18	373.25 ± 32.24	127.33 ± 22.24
	Observation group	62.75 ± 21.26	57.63 ± 12.32	1.25 ± 0.32	315.91 ± 32.02	117.23 ± 20.57

[2]	Comparison group	71.34 ± 13.25	49.62 ± 12.31	1.64 ± 0.25	373.27 ± 31.07	123.24 ± 24.25
	Observation group	67.33 ± 22.24	56.31 ± 12.81	1.33 ± 0.24	304.30 ± 31.19	113.25 ± 24.24

[13]	Comparison group	77.23 ± 10.57	40.30 ± 2.19	1.63 ± 10.57	376.67 ± 13.24	125.91 ± 13.02
	Observation group	67.24 ± 14.53	57.63 ± 2.32	1.24 ± 14.53	303.23 ± 12.26	113.27 ± 17.07

[5]	Comparison group	77.34 ± 10.18	44.34 ± 3.25	1.64 ± 10.18	363.76 ± 21.15	124.30 ± 21.19
	Observation group	69.26 ± 10.63	52.33 ± 3.24	1.26 ± 10.63	312.75 ± 21.26	117.33 ± 21.24

## Data Availability

The experimental data used to support the findings of this study are available from the corresponding author upon request.
